# Noncontact ECG Monitoring by Capacitive Coupling of Textiles in a Chair

**DOI:** 10.1155/2021/6698567

**Published:** 2021-06-16

**Authors:** Po-Cheng Su, Ya-Hsin Hsueh, Ming-Ta Ke, Jyun-Jhe Chen, Ping-Chen Lai

**Affiliations:** ^1^Department of Electronic Engineering, National Yunlin University of Science and Technology, Douliu 64002, Taiwan; ^2^Bachelor Program in Intelligent Robotics, National Yunlin University of Science and Technology, Douliu 64002, Taiwan

## Abstract

Some patients are uncomfortable with being wired to a device to have their heart activity measured. Accordingly, this study adopts a noncontact electrocardiogram (ECG) measurement system using coupled capacitance in a conductive textile. The textiles can be placed on a chair and are able to record some of the patient's heart data. Height and distance between the conductive textile electrodes were influential when trying to obtain an optimal ECG signal. A soft and highly conductive textile was used as the electrode, and clothing was regarded as capacitance insulation. The conductive textile and body were treated as the two electrode plates. This study found that placing the two conductive textiles at the same height provided better data than different heights. The system also enabled identifying the P, Q, R, S, and T waves of the ECG signal and eliminated unnecessary noise successfully.

## 1. Introduction

Electrocardiogram (ECG) health monitors are often applied directly to the body. The standard procedure involves the use of a 12-lead connection in a controlled hospital environment. However, in some situations, such as during exercise, while driving, or when a person is considered a high-risk patient, accurate real-time ECG data would be helpful but cannot be obtained.

ECG technological studies cover many engineering fields. For example, noncontact ECG measurement approaches include radar [1], printed circuit boards (PCBs) electrodes [2], imaging devices [3], and others more [4, 5]. One such study by Ritchie et al. [6] researched fire-fighters, continuously monitoring their physiological signals through a noncontact metal electrode sensor system with wireless communication.

In noncontact or indirect ECG measurements, conductive textiles are used in wearable devices, like those found in Castro et al. [7], where a capacitive coupling-based ECG used noncontact evaluation methods to assess sleep apnoea cases. The device functioned by intercepting the signals given by various positions in controlled sleep environments. Yu [8] created a different nonintrusive ECG sensor. A steering wheel contained the necessary electrodes, and that sensor could then log the participant's heart rate variability during a two-hour driving simulation. Currently, if the conductive fibres are embedded or woven into fabrics, the electrical conductivity deteriorates after washing. Thus far, conductive fibres used in such cases have all suffered the same shortcoming.

Silva et al. [5] also proposed various types of conductive textiles as an interface between the skin and the sensor and collected data to evaluate and produce a correlative index. Lim et al. [2] employed PCB electrodes for a seated participant that could take ECG readings through test participants' clothes. The different types of cloth, such as cotton, wool, and acrylic, all caused differing frequency responses, showing that if the material is worn, it significantly impacted readings. Rachim and Chung [4] adopted a technique of capacitive-coupled electrodes, measuring physiological signals through clothes. The method also enabled the detection of ECG signals through the arms via a wearable device. Although the signals from the arms were weak and there was significant noise, the signal was sufficient for analysis. Even when tested with various thicknesses of clothes, the signals were detectable.

This paper proposes an alternate ECG data detection system. Conductive textiles have the advantage of being soft and fitting the human body well. Using these textiles, this novel noncontact ECG detection system adapts these materials for use in a chair to measure ECG data. The system could be used in a chair, car seat, mattress, or countless other products. The data obtained by the test system could be used for the provision of medical or safety services such as measurement of fatigue while driving, monitoring the elderly, and so on.

## 2. Methods

### 2.1. Principles of Noncontact ECG Monitoring

This study uses capacitive coupling to measure a participant's ECG data using noncontact methods [9]. However, the high input impedance of an operational amplifier means that the system has a high sensitivity. At the input stage, external noise such as power lines may generate incorrect data. For this reason, it is necessary to shield the device from an isolating material. The shielding layer must be earthed to give a path for the noise to follow, which it will do because of the low impedance. Furthermore, stray capacitances exist between the sensing and shielding layers due to the electric potential difference. As a result, the operational amplifier's function eliminates power line noises and decreases signal interference.

The capacitance sensing principle is extended with a capacitive-coupled electrode [8]. The capacitance feature mainly allows an alternating signal to pass through it to achieve the required coupling signal function. The conductive textile is regarded as a parallel plate in this capacitive-coupled electrode (Figure 1). The body is considered the other parallel capacitance plate, and clothes are treated as a capacitance insulation layer. A physiological signal will be inducted into the circuit by this capacitance.

### 2.2. Electrocardiogram Measurements

We adopted a commercial ECG module (Raising Technology Co., Ltd, Taiwan). The sample rate was 250 Hz, and electrocardiographic patches were attached to a patient's chest at specific locations to the chest lead. In this ECG module, the band-pass filter was set in the range 1–194 Hz, where 1 Hz was the cut-off frequency of the high-pass filter, and 194 Hz was the cut-off frequency of the low-pass filter. The tested system uses the adopted amplifier circuit to amplify the ECG signals to a gain of between 100 and 1000 times.

### 2.3. Configuration of Conductive Textiles

Two sheets of the conductive textile (7  cm × 5  cm) were configured on the back of a chair as a sensing electrode, and a sheet of conductive textile (21  cm × 29.7  cm) was placed on the seat as shown in Figure 2.

In this set-up, the capacitive-coupled electrodes behaved similarly to resistors and were connected in parallel. From equivalent circuit elements, the coupling impedance *Z* of the capacitive-coupled electrode can be determined by

(1) $$\begin{array}{c} Z=\;\frac{R_{1}}{\sqrt{1+{\left(2\pi fR_{1}C_{1}\right)}^{2}}}=\;\frac{1}{\sqrt{\left(1/R_{1}^{2}\right)+{\left(2\pi fC_{1}\right)}^{2}}}, \end{array}$$

where *C*_1_ is the equivalent capacity of the capacitive-coupled electrode; *R*_1_ is the equivalent electrical resistance of the capacitive-coupled electrode, and *f* is the equivalent supply frequency of the capacitive-coupled electrode. As the equivalent electrical resistance *R*_1_ approaches infinity in this situation, the equation resolves to the form shown in

(2) $$\begin{array}{c} Z=\frac{1}{2\pi fC_{1}}. \end{array}$$

Equivalent capacitance *C*_1_ can be determined by the

(3) $$\begin{array}{c} C_{1}=\;\varepsilon_{0}\varepsilon_{r}\frac{A}{d}, \end{array}$$

where *ε*_0_*ε*_*r*_ is the dielectric coefficient (*ε*_0_ being vacuum permittivity; *ε*_*r*_ being the dielectric constant of cloth), *A* is the area of the capacitive coupling, which indicates the effective contact area of conductive textiles, and *d* is the distance of that capacitor (i.e., the distance between the conductive textile and the body is equivalent to the thickness of the clothing). Then, the impedance *Z* can be determined by equation (4) below:

(4) $$\begin{array}{c} Z=\frac{1}{2\pi f}\times \frac{1}{\varepsilon }\times \frac{d}{A}. \end{array}$$

Accordingly, as the distance between the conductive textiles and body becomes less or the effective contact area becomes greater, the impedance becomes smaller. The signal is more easily transmitted.

This paper utilizes a conductive textile area of “*A*  = 35 cm^2^ (5 cm × 7 cm),” “*d*  = 0.12 mm,” and “*ε*_*r*_  = 1”, meaning that the coupling capacitance follows

(5) $$\begin{array}{c} C_{1}=\varepsilon_{0}\varepsilon_{r}\frac{A}{d}=258.13pF. \end{array}$$

### 2.4. Measurement Results

The commercial ECG module is composed of a driven-right-leg circuit, second-order high-pass filter, 60-Hz band-rejection filter, and a second-order low-pass filter in the filter and amplifying unit. The band-pass filter is 1 Hz to 194 Hz. The participant's height was 182 cm, weight was 80 kg, and the participant was wearing clothes made of 100% cotton. The participant sat on the measurement chair for estimation. The participant was asked to wear 100% cotton clothes as this would produce less static electricity, and electrostatic discharges (ESDs) may affect the device measurements. The noncontact ECG signal noise was greater than direct contact ECG signals, as shown in Figure 3. Therefore, further investigation was conducted into the optimization of positions of the conductivity textiles.

As expected, and as shown in Equation (4), ECG signal detection was affected by the distance between the conductive textile and body and the effective contact area of the conductive textile. In previous studies [2, 7], the researcher addressed this issue by adapting the conductive textile itself. However, the relation between different placement locations of the conductive textiles has not been investigated. Therefore, this study also analyses the placement of the conductive textiles regarding ECG signal detection. Five configured placement methods were tested and are shown in Table 1. Electrode placement was at or near the lower margin of the heart. On the participant, this was a height of approximately 35 cm from the seat, as shown in Figure 4. Measurement locations selected detail the lowest level of the electrode, i.e., from 31 cm height, extending upward, and 27 cm height extending upward. The actual height is approximately 31 cm when measured from the seat, as shown in Figure 2, and the electrodes placed near the heart, as shown in Figure 5. It presents the relative position of a seated participant. Note that there is an incline between the body and the chair due to natural posture. Regarding the cushion as the base, the electrode is 31 cm, the centre of which is 31 + 3.5 cm (the electrode's length is 7 cm). When the participant is seated, there was an elevation difference caused by the slope between the heart's lower margin and the electrode position.

We detected the ECG signals. The sampling rate was 250 Hz using conductive textile as electrodes were then digitally low-pass filtered at cut-off frequencies of 30 Hz. We calculated signal-to-noise ratio (SNR) for each experiment using Matlab software to compare the ECG signal-measuring performance using conductive textile in different detecting places. The SNR of ECG signals [11], as the ratio of the ECG to the noise power in 10 s, is defined as follows:

(6) $$\begin{array}{c} \text{SNR}=10\;\log_{10}\left(\frac{\sum_{n=1}^{N}f{\left(n\right)}^{2}}{\sum_{n=1}^{N}{\left[\left|f\left(n\right)-\hat{f}\left(n\right)\right|\right]}^{2}}\right), \end{array}$$

where *f*(*n*) is an ECG signal containing noise, $\hat{f}\left(n\right)$ is the signal denoising with low-pass filtered at cut-off frequencies of 30 Hz, and N is the length of the signal.

The original ECG signals measured from experiments 1 to 6 are shown in Figures 6–11 . In experiment 1, the height is 31 cm, left and right sides both 8 cm lateral from the midline. The voltage of R peak is 2.16 V. In experiment 2, the electrodes were placed at the height of 31 cm, left side 4 cm lateral from the midline and right side 8 cm lateral. The voltage of R peak is 2.08 V. In experiment 3, the position of electrodes was at 31 cm height, left and right sides 4 cm lateral from the midline. The voltage of R peak can reach 1.84 V. In experiment 4, the height is 31 cm, left side 8 cm lateral from the midline and right side 4 cm lateral. The voltage of R peak is 2.16 V. In experiment 5, the electrodes were placed left 27 cm height and right 31 cm height, left and right sides both 8 cm lateral from the midline. The voltage of R peak reaches 0.232 V. In experiment 6, the position of electrodes was at 27 cm height, left and right sides both 8 cm lateral from the midline with the voltage of R peak 0.232 V. After we got the signal, we calculated the SNR. The SNR of the measured signal is shown in Table 2.

## 3. Discussion

In experiments 1, 2, 3, and 4, the two conductive textiles' height on both the left and right sides were 31 cm. The ECG signal indicated that the signal-to-noise ratio (SNR) in experiments 1, 2, 3, and 4 were similar. This caused the electrode detection area to exceed the width of the participant's back, reducing the effective contact area. As the effective area declined, the coupling capacitance value rose. The cut-off frequency for the capacitance input impedance *R*_*Bias*_ that forms the high-pass filter increases; thus, the signal decreases. Furthermore, it can be observed from Figures 6 and 8 that there exists a positive correlation between the signals in experiments 1 and 3, which concerns the lateral distance of the conductive textiles. The device received considerably clearer ECG signals when the distance was closer between the two conductive textiles and the placement was closer to the heart. Experiment 2 and experiment 4 show that when the distance between the conductive textiles was 12 cm, it was much closer to the heart (Figures 7 and 9). The SNR of the measured signal was approximately 24.22 and 24.62, which is higher than the amplitude observed in experiment 1 (24.00).

The lateral placement of the conductive textiles and the height have a significant impact on ECG signals detection. In experiments 1 to 4, the lateral distance of both the left and right conductive textiles was particularly insignificant. The height of the conductive textiles sometimes differed; for example, in experiment 1, both textiles were placed at 31 cm, whereas in experiment 5, both were placed at 27 cm.  Figure 10 shows the results of experiment 5. Taking the body length of this particular participant as an example, 31 cm represents the position closest to the fifth rib as it extends from the vertebrae. 27 cm was below the fifth rib when the participant was seated. For a person of the participant's size, the heart is approximately 35 cm above the seat and 30 cm from the cushion. As a result, the sensor height of 31 cm is the optimal position for ECG measurement.

Experiments 1, 4, and 5 all involved conductive textile pads positioned 8 cm laterally from the participant's midline. Figures 10 and 11 show the results of experiments 5 and 6. The outcome from experiment 1 is better than the others; even though the ECG signals suffer from noise interference. The Q, T, and U wave can still be detected in the ECG signal. This outcome is caused by the position of the two electrodes, particularly the height factor. Compared to experiments 4 and 5, when the left electrode is moved down to 27 cm, the width of the coupling capacitance exceeds the original preset value (*d* = 0.12 mm), and the sensing position moves away from the heart. Furthermore, the electric current generated when the myocardium is active is not easily measured. Simultaneously, the ascent or descent of the rib during breathing causes the body to move slightly, resulting in significant amounts of noise being measured in the ECG readings.

## 4. Conclusions

This study uses flexible conductive fibres as an intermedium and achieves noncontact ECG signal measurement. Where the participant remains seated and without interference, the ECG pattern can detect and record. This study treated clothes as a capacitance insulator and used the conductive textile and body as a pair of electrode plates so that capacitive coupling properties could be used to determine an ECG signal.

Primary signal processing was undertaken by a differential amplifier, which passed the signal through a two-level high-pass filter and a two-level low-pass filter, sequentially. Thus, the ECG signal was obtained from the ECG module. Some literature has shown that recording ECG signals using capacitive coupling electrodes in noncontact situations is possible, but the system included electrodes or involved direct contact and made users feel uncomfortable [8, 12, 13].

This study showed that during noncontact measurement techniques with conductive textiles the waveform result is closely related to the location of the capacitance textiles. Upper body length, back width, habitual sitting posture, and breathing all affect readings. The experiment result demonstrates that the waveform obtained by this method may cause the P, Q, R, S, and T waves to become indistinguishable. In addition, we discover that these two electrodes when positioned at the same height are better than at different heights. However, even given an inappropriate position, the R wave can still be identified. As a result, applied correctly, the system can still use noncontact methods to calculate heart rate, the R-R interval of HRV, and other derivative items.

## Figures and Tables

**Figure 1:** Schematic diagram of the proposed capacitance model [10].

**Figure 2:** Photograph of conductive textile configuration.

**Figure 3:** Comparison of (a) noncontact ECG measurement and (b) direct contact with body ECG measurement.

**Figure 4:** Profile view of the participant and device relative positions.

**Figure 5:** Rear aspect view of the participant measurement position.

**Figure 6:** Experiment 1, 31 cm height, left and right sides both 8 cm lateral from the midline.

**Figure 7:** Experiment 2, 31 cm height, left side 4 cm lateral from the midline and right side 8 cm lateral.

**Figure 8:** Experiment 3, 31 cm height, left and right sides 4 cm lateral from the midline.

**Figure 9:** Experiment 4, 31 cm height, left side 8 cm lateral from the midline and right side 4 cm lateral.

**Figure 10:** Experiment 5, left 27 cm height and right 31 cm height, left and right sides both 8 cm lateral from the midline.

**Figure 11:** Experiment 6, 27 cm height, left and right sides both 8 cm lateral from the midline.

**Table 1:** Conductive textile placement configuration table for tests at two heights and distances from seated participant midline.

Expt.	Right side placement	Left side placement
1	8 cm lateral, 31 cm height	8 cm lateral, 31 cm height
2	8 cm lateral, 31 cm height	4 cm lateral, 31 cm height
3	4 cm lateral, 31 cm height	4 cm lateral, 31 cm height
4	4 cm lateral, 31 cm height	8 cm lateral, 31 cm height
5	8 cm lateral, 31 cm height	8 cm lateral, 27 cm height
6	8 cm lateral, 27 cm height	8 cm lateral, 27 cm height

**Table 2:** The SNR of measured signal for each experiment.

Experiment	Expt. 1	Expt. 2	Expt. 3	Expt. 4	Expt. 5	Expt. 6
SNR	24.00	24.22	25.02	24.62	15.06	15.02

## Data Availability

All the data are already given in the manuscript.

## References

[1] Yang X., Sun G., Ishibashi K. Non-contact acquisition of respiration and heart rates using Doppler radar with time domain peak-detection algorithm.

[2] Lim Y. G., Kim K. K., Park K. S. (2006). ECG measurement on a chair without conductive contact. *IEEE Transactions on Biomedical Engineering*.

[3] Lewandowska M., Rumiński J., Kocejko T., Nowak J. Measuring pulse rate with a webcam — A non-contact method for evaluating cardiac activity.

[4] Rachim V. P., Chung W.-Y. (2016). Wearable noncontact armband for mobile ECG monitoring system. *IEEE Transactions on Biomedical Circuits and Systems*.

[5] Silva H., Lourenco A., Leite P., Coutinho D., Fred A. Study and evaluation of a single differential sensor design based on electro-textile electrodes for ECG biometrics applications.

[6] Ritchie P., Huerta M., Lau T. L., Agee J., Cao H., Chiao J. C. Passive continuous electrocardiogram monitoring of firemen using non-contact electrodes.

[7] D Castro I., Varon C., Torfs T. (2018). Evaluation of a multichannel non-contact ECG system and signal quality algorithms for sleep Apnea detection and monitoring. *Sensors*.

[8] Yu X. (2009). Real-time nonintrusive detection of driver drowsiness. *Technical Report*.

[9] Lopez A., Richardson P. C. (1969). Capacitive electrocardiographic and bioelectric electrodes. *IEEE Transactions on Biomedical Engineering*.

[10] Ueno A., Uchikawa Y., Noshiro M. A capacitive sensor system for measuring laplacian electromyogram through cloth: a pilot study.

[11] Ai Q., Liu Q., Meng W., Xie S. Q. Neuromuscular signal acquisition and processing.

[12] Hou Z., Dong Y., Wu X. (2020). A template Addition method for eigentriple rearrangement in singular spectrum analysis for processing biopotential signals with extremely lower SNRs. *IEEE Sensors Journal*.

[13] Wang T.-W., Zhang H., Lin S.-F. (2020). Influence of capacitive coupling on high-fidelity non-contact ECG measurement. *IEEE Sensors Journal*.

